# Nitric Oxide Inhalation Therapy Attenuates Postoperative Hypoxemia in Obese Patients with Acute Type A Aortic Dissection

This article has been retracted.

**DOI:** 10.1155/2022/9612548

**Published:** 2022-03-22

**Authors:** Ping Zheng, Dingsheng Jiang, Chun Liu, Xiang Wei, Shiliang Li

**Affiliations:** Department of Cardiothoracic and Vascular Surgery, Tongji Hospital, Tongji Medical College, Huazhong University of Science and Technology, Wuhan, Hubei 430030, China

## Abstract

**Objective:**

To investigate the differences between inhaled nitric oxide (iNO) treatment and conventional therapy in the treatment of postoperative hypoxemia in obese patients with acute type A aortic dissection (ATAAD).

**Methods:**

ATAAD patients diagnosed and treated with emergency surgery in our hospital from June 2017 to December 2019 were retrospectively analyzed. Patients with postoperative hypoxemia were divided into the iNO group and control group. Propensity score matching was used to analyze clinical characteristics and results of the two groups.

**Results:**

A total of 218 ATAAD patients with BMI ≥ 25 were treated with surgery. Among them, 115 patients developed refractory hypoxemia (64 in the control group and 51 in the iNO group). Patients in the iNO group had significantly shorter invasive mechanical ventilation time, intensive care unit (ICU) stay, and hospital stay. After 6 h of iNO treatment, the PaO_2_/FiO_2_ ratio in the iNO group increased significantly, and this ratio was higher than that in the control group at 6, 12, 24, 48, and 72 h after treatment.

**Conclusion:**

Low-dose iNO could improve oxygenation and shorten mechanical ventilation and ICU stay in patients with hypoxemia after ATAAD surgery, but without significant side effects or increase in postoperative mortality or morbidity. These findings provide a basis for a randomized multicenter controlled trial to assess the efficacy of iNO in the treatment of hypoxemia after ATAAD surgery.

## 1. Introduction

Acute aortic dissection (AAD) is one of the most serious cardiovascular diseases, with dangerous conditions, a high mortality rate, and an annual prevalence of approximately 3/100,000 [1, 2]. According to Stanford classification, AAD can be divided into type A and type B; acute type A aortic dissection (ATAAD) accounts for about 65% of AAD, which involves the ascending aorta. Surgery can save the lives of most ATAAD patients, but postoperative morbidity is still high which ranges from 9% to 30% [3–5]. Hypoxemia occurs following destruction of aortic vascular tissue, intraoperative cardiopulmonary bypass (CPB), ischemia/reperfusion injury, massive transfusion, deep hypothermia, and occurs secondary to systemic and local inflammatory responses [6–9]. A Chinese study has shown that postoperative hypoxemia is a serious complication after ATAAD with an incidence of approximately 30-50%, which is defined as the ratio of arterial oxygen partial pressure to fractional inspired oxygen (PaO_2_/FiO_2_) ≤ 200 mmHg within 24 h after surgery [10]. Foreign studies have shown a similar conclusion, and found that hypoxemia not only prolongs the postoperative mechanical ventilation time and ICU stay of AAD patient, but also increases the perioperative mortality rate [11]. Additionally, long-term postoperative hypoxemia can cause functional damage to other organs except the lungs, affecting postoperative long-term survival [12]. However, effective medical interventions for this disease are limited and controversial [13].

Inhaled nitric oxide (iNO) is a selective pulmonary vasodilator that has long been used to treat acute respiratory distress syndrome (ARDS), pulmonary hypertension, neonatal hypoxic respiratory failure, and lung transplantation. Some randomized controlled trials and analyses have so far proved that iNO treatment has no benefit on mortality and duration of mechanical ventilation in ARDS patients [14, 15]. However, there are differences in etiology and pathophysiology between hypoxemia after ATAAD surgery and ARDS. It has previously been found that iNO improves oxygenation after AAD and shortens extubation time [16]. This study retrospectively compared the efficacy and safety of low-dose iNO therapy with traditional treatment for hypoxemia after AAD surgery because of the lack of randomized controlled or case-control studies on this field.

## 2. Materials and Methods

### 2.1. Study Subjects

Patients who were diagnosed with ATAAD and underwent emergency surgery in our hospital from June 2017 to December 2019 were retrospectively analyzed. The included patients were divided according to the treatment method: conventional treatment patients (control group) and iNO-treated patients (iNO group). This study was approved by the Ethics Committee of Tongji Medical College of Huazhong University of Science and Technology (Approval no. TJ-IRB20210962).

Inclusion criteria were as follows: (1) patients diagnosed with ATAAD by multislice computed tomography and color Doppler ultrasonography; (2) patients who underwent repair surgery, including ascending aortic replacement (AAR), total arch replacement (TAR), and elephant trunk stent; (3) patients with a body mass index (BMI) ≥ 25; and (4) patients with postoperative refractory hypoxemia (PaO_2_/FiO_2_ ≤ 200 mmHg), and within 6 hours after ICU admission, this value was still ≤100 mmHg despite conventional treatment.

Exclusion criteria were as follows: (1) patients with reoccurrence; (2) patients who did not undergo cardiac surgery, such as patients who died before surgical intervention; (3) patients who died within 24 h after repair surgery; (4) patients with chronic inflammation, lung cancer, emphysema, tuberculosis, or connective tissue disease; (5) patients with serious postoperative complications, such as coma, cardiogenic shock, and gastrointestinal ischemia; (6) patients with postoperative complications such as stroke or spinal cord injury which may lead to respiratory failure; and (7) patients with severe cognitive impairment or language problems.

### 2.2. Treatment Methods

#### 2.2.1. Conventional Treatment

This includes (1) optimization of mechanical ventilation settings, including tidal volume regulation and positive end-expiratory pressure (PEEP) titration; (2) chest drainage for pleural effusion or pneumothorax; (3) optimization of fluid management; and (4) intravenous injection of 40 mg prednisolone and 300,000 units of ulinastatin for 3 consecutive days, twice daily.

#### 2.2.2. iNO Therapy

Patients with refractory hypoxemia were treated with 5-10 ppm iNO. After successful extubation, iNO could be administered via nasal cannula and ended by tapering the flow over 24 h. The total treatment procedure ended if the PaO_2_/FiO_2_ ratio was as high as 150 mmHg after 2 to 6 h of iNO withdrawal.

#### 2.2.3. Extubation Criteria

The criteria were as follows: (1) patients with a clear state of consciousness and appropriate muscle strength; (2) patients with hemodynamic stability and with no signs of low cardiac output syndrome or myocardial ischemia, who required little positive inotropic support; (3) thoracic catheter drainage < 50 mL/h, without active bleeding; (4) sufficient oxygenation; (5) successful daily spontaneous breathing test (SBT); and (6) without severe anxiety or diaphoresis.

### 2.3. Clinical Results

#### 2.3.1. General Information of Patients

The following information of patients were recorded: age, gender, BMI, smoking history, hypertension, diabetes mellitus, chronic obstructive pulmonary disease, cerebrovascular events, myocardial infarction, pericardial effusion, lower limb ischemia, and aortic regurgitation.

#### 2.3.2. Laboratory Test Results

Laboratory tests were performed within 1 h after diagnosis, including serum triglyceride (TG), total cholesterol (TC), high-density lipoprotein cholesterol (HDL-c), white blood cell count (WBC), platelet (PLT), alanine aminotransferase (ALT), and creatinine (Cr).

#### 2.3.3. Surgical Indicators

First, preoperative PaO_2_/FiO_2_ of patients and the time from onset to surgery were collected. Then, characteristics of patients during surgery were recorded, mainly including CPB time, deep hypothermic circulatory arrest (DHCA) time, aortic cross-clamping time, minimum rectal temperature, 24 h blood transfusion, and PaO_2_/FiO_2_ ratio. Additionally, the PaO_2_/FiO_2_ ratio was also collected after surgery and within 72 h after iNO treatment for refractory hypoxemia.

#### 2.3.4. Postoperative Outcomes

The following outcome measures were collected: postoperative death, duration of invasive mechanical ventilation, intensive care unit (ICU) stay, length of hospital stay, drainage volume within 72 h after iNO therapy, sudden cardiac arrest, pulmonary infection, septicemia, thrombocytopenia, and acute renal failure.

### 2.4. Statistical Analysis

Data analysis was performed using SPSS 21.0 software (IBM Corp., Armonk, NY, USA). Continuous data with normal distribution were presented as mean ± standard deviations (SD) and compared with the *t*-test. Enumeration data were expressed as percent (%) and compared using the *χ*^2^ test. *P* < 0.05 was the criterion for statistically significant differences.

## 3. Results

### 3.1. Preoperative Clinical Characteristics

In this study, 218 ATAAD patients with BMI ≥ 25 underwent surgery. Then, patients' postoperative death and serious complications were excluded, and therefore, 115 patients who experienced postoperative refractory hypoxemia were finally included in our trial. They were divided into a control group (*n* = 64, conventional treatment) and iNO group (*n* = 51, iNO therapy). The preoperative clinical characteristics of patients are shown in Table 1, and no significant statistical difference was found in all included parameters, providing assurance of comparability.

### 3.2. Intraoperative Clinical Characteristics

The clinical characteristics of the two groups during surgery are summarized in Table 2. No significant differences were identified between the control and iNO groups in CPB time, DHCA time, aortic cross-clamping time, minimum rectal temperature, 24 h blood transfusion volume, and PaO_2_/FiO_2_ ratio.

### 3.3. Postoperative Clinical Characteristics

There was no marked difference in the PaO_2_/FiO_2_ ratio between the two groups after surgery when refractory hypoxemia occurred. However, after 6 h of iNO treatment, the PaO_2_/FiO_2_ ratio in the iNO group was significantly increased, and this ratio was higher than that in the control group at 6, 12, 24, 48, and 72 h after iNO treatment (Figure 1).

The postoperative clinical characteristics of patients in the control and iNO groups are shown in Table 3. In general, no marked differences were identified between the two groups in mortality, drainage volume within 72 h after iNO therapy, sudden cardiac arrest, pulmonary infection, septicemia, thrombocytopenia, and acute renal failure. However, in comparison with those in the control group, patients in the iNO group had significantly shorter invasive mechanical ventilation time, ICU stay, and hospital stay (*P* < 0.05).

## 4. Discussion

We investigated the efficacy and safety of iNO in the treatment of postoperative hypoxemia in ATAAD patients through a retrospective case-control study. The results indicated that iNO treatment in patients with refractory hypoxemia after ATAAD surgery was associated with improved arterial oxygenation and shorter invasive mechanical ventilation time.

Hypoxemia is a common complication after cardiothoracic surgery [17] with an incidence of about 7% [18], but the incidence increases to 50.88% after ATAAD surgery [19]. Patients with postoperative hypoxemia often require prolonged mechanical ventilation [20]. According to previous studies, postoperative hypoxemia in ATAAD patients is associated with multiple risk factors, including prolonged CPB, aortic root occlusion, DHCA, lung injuries, and excessive inflammatory response [21–23]. iNO can rapidly lead to ventilation/perfusion matching and then improve oxygenation of the damaged lung. Rossaint et al. [24] first reported in 1993 that iNO treatment could improve oxygenation in ARDS patients. Subsequent studies have shown that similar improvements in oxygenation do not have better results in a dose-dependent manner [15]. Several systematic reviews have revealed that there is no relation of iNO with the reduction in mortality and in the duration of mechanical ventilation in ARDS patients, while iNO treatment may even increase the incidence of renal impairment [14]. However, low-dose iNO (<5 ppm) has been proved to improve lung function at 6 months in ARDS survivors [25]. In general, iNO dilates the blood vessels of ventilated alveoli and increases their blood flow, thereby counteracting ventilation/perfusion mismatch [14]. These previous studies inspired us to explore whether iNO therapy has potential efficacy on refractory hypoxemia after ATAAD surgery [26–28]. In recent years, it has been found that iNO reduces intrapulmonary shunts and increases the PaO2/FiO2 ratio in postoperative ATAAD patients, thereby improving severe hypoxemia [29]. In the present study, we found that iNO treatment did consistently improve oxygenation in patients with refractory hypoxemia within 72 hours, with a higher PaO_2_/FiO_2_ ratio in the iNO group. Zhang et al. [30] similarly confirmed that low doses of iNO improved oxygenation in patients with hypoxemia after ATAAD surgery. So far, the mechanism for the relation between hypoxia and ATAAD surgery is unclear. In this study on refractory hypoxemia, we excluded common hypoxemia-related pathologies such as sputum obstruction, interstitial pulmonary edema, or extrapulmonary changes by clinical observations, radiographs, and lung ultrasound. And we therefore supposed that the underlying mechanism of refractory hypoxemia after ATAAD surgery may be attributed to intrapulmonary shunting caused by an excessive inflammatory response. The clinical effect of iNO in the treatment of refractory postoperative hypoxemia in this study may indirectly support our hypothesis.

Collectively, in comparison with the conventional therapy, iNO treatment led to improvement in oxygenation and consequently the reduction in invasive mechanical ventilation duration, ICU stay, and hospital stay. And patients could receive iNO treatment even after extubation and ventilator weaning. However, this therapy did not improve mortality, which was similar to the results of other studies [30, 31]. Additionally, it should be noted that a higher dose of iNO was not given, because the clinical efficacy was relatively satisfactory at a dose of 5 ppm and no adverse reactions occurred.

There were limitations in this study: (1) more clinical analysis indicators should be included, such as treatment costs, treatment efficacy, and safety; (2) the sample size needs to be further expanded; and (3) there is missing information on postoperative follow-up of patients.

## 5. Conclusion

This retrospective analysis suggests that iNO may be considered a treatment for patients with refractory hypoxemia after ATAAD surgery. This approach may lead to a continuous improvement in oxygenation and a reduction in the duration of invasive mechanical ventilation. Future studies are still required to optimize the clinical implementation of iNO and to further elucidate the pathogenesis of hypoxemia after ATAAD surgery.

## Figures and Tables

**Figure 1:** PaO_2_/FiO_2_ ratio before surgery, after surgery, and within 72 h after iNO treatment in the two groups. Data were presented as mean ± standard deviations (SD). ^∗^*P* < 0.05*vs*. control group.

**Table 1:** Preoperative clinical characteristics of patients in the two groups.

Variables	Control group (*n* = 64)	iNO group (*n* = 51)	*χ* ^2^/*t*	*P*
Baseline characteristics				
Age (years)	52.67 ± 7.53	54.16 ± 7.93	-1.027	0.307
BMI (kg/m^2^)	26.69 ± 2.71	26.97 ± 3.46	-0.456	0.650
Male gender	43 (67.2)	34 (66.7)	0.003	0.953
Current smoking	32 (50.0)	27 (52.9)	0.098	0.754
Hypertension	45 (70.3)	37 (72.5)	0.069	0.792
Diabetes	3 (4.7)	4 (7.8)	0.494	0.482
Pericardial effusion	6 (9.4)	5 (9.8)	0.006	0.938
Ischemic stroke induced by ATAAD	3 (4.7)	2 (3.9)	0.040	0.841
Lower limb ischemia	0 (0.0)	1 (2.0)	1.266	0.261
Aortic regurgitation	12 (18.8)	14 (27.5)	1.228	0.268
Mesenteric ischemia	2 (3.1)	2 (3.9)	0.054	0.817
Laboratory tests				
TG (mmol/L)	2.22 ± 0.47	2.16 ± 0.41	0.749	0.455
HDL-c (mmol/L)	103.70 ± 17.06	105.57 ± 17.07	-0.582	0.561
WBC (10^9^/L)	10.62 ± 2.81	10.22 ± 2.36	0.815	0.417
PLT (10^9^/L)	201.30 ± 41.09	200.26 ± 32.56	0.147	0.883
Cr (*μ*mol/L)	133.81 ± 29.87	140.02 ± 28.55	-1.129	0.261
ALT (U/L)	172.04 ± 28.76	177.65 ± 36.22	-0.902	0.370
Preoperative PaO_2_/FiO_2_ rate (mmHg)	275.79 ± 58.54	284.24 ± 26.54	-0.780	0.437

Data are mean ± SD or *n* (%). BMI: body mass index; ATAAD: acute type A aortic dissection; TG: triglyceride; TC: total cholesterol; HDL-c: high-density lipoprotein cholesterol; WBC: white blood cell count; PLT: platelet; Cr: creatinine; ALT: alanine aminotransferase; PaO_2_/FiO_2_: arterial oxygen partial pressure/fractional inspired oxygen.

**Table 2:** Intraoperative clinical characteristics of patients in the two groups.

Variables	Control group (*n* = 64)	iNO group (*n* = 51)	*t*	*P*
Minimum rectal temperature (°C)	25.31 ± 4.23	26.37 ± 3.07	-1.555	0.123
CPB time (min)	336.89 ± 44.17	349.63 ± 54.66	-1.382	0.170
Aortic cross-clamping time (min)	153.14 ± 31.97	164.90 ± 36.87	-1.801	0.075
DHCA time (min)	28.38 ± 7.43	30.65 ± 6.04	-1.764	0.080
Transfusion volumes of RBCs (U)	5.95 ± 1.19	6.37 ± 1.51	-1.624	0.108

Data are mean ± SD. CPB: cardiopulmonary bypass; DHCA: deep hypothermic circulatory arrest.

**Table 3:** Postoperative clinical characteristics of patients in the two groups.

Variables	Control group (*n* = 64)	iNO group (*n* = 51)	*χ* ^2^/*t*	*P*
Mortality	4 (6.3)	3 (5.9)	0.007	0.935
Duration of invasive mechanical ventilation support (h)	127.48 ± 21.57	72.82 ± 13.94	16.421	≤0.001
Noninvasive ventilation support requirements	18 (28.1)	19 (37.3)	1.084	0.298
Pulmonary infections	0 (0.0)	0 (0.0)	—	—
Bloodstream infections	0 (0.0)	0 (0.0)	—	—
Surgical site infections	2 (3.1)	1 (2.0)	0.151	0.697
AKI	22 (34.4)	19 (37.3)	0.103	0.749
Postoperative drainage within 72 h (mL)	1548.96 ± 292.68	1470.28 ± 166.08	1.815	0.072
Length ICU stay (days)	13.63 ± 2.61	8.76 ± 3.02	9.246	≤0.001
Length of hospital stay (days)	23.47 ± 3.15	19.82 ± 4.20	5.151	≤0.001

## Data Availability

The datasets supporting the conclusions of this article are included within the article.

## Abbreviations

iNO: Inhaled nitric oxide
ATAAD: Acute type A aortic dissection
PSM: Propensity score matching
AAD: Acute aortic dissection
CPB: Cardiopulmonary bypass
AAR: Ascending aortic replacement
TAR: Total arch replacement
BMI: Body mass index
PEEP: Positive end-expiratory pressure
SBT: Spontaneous breathing test
TG: Triglyceride
TC: Total cholesterol
HDL-c: High-density lipoprotein cholesterol
WBC: White blood cell count
PLT: Platelet
ALT: Alanine aminotransferase
Cr: Creatinine
DHCA: Deep hypothermic circulatory arrest.
